# Asymmetric effects of foreign direct investment and globalization on ecological footprint in Indonesia

**DOI:** 10.1371/journal.pone.0297046

**Published:** 2024-01-26

**Authors:** Hung Van Tran, Anh Viet Tran, Ngoc Bui Hoang, Tram Nguyen Huynh Mai

**Affiliations:** 1 Hung Vuong University of Ho Chi Minh City, Ho Chi Minh City, Vietnam; 2 Faculty of Business Administration, Ho Chi Minh City University of Industry and Trade, Ho Chi Minh City, Vietnam; 3 Ho Chi Minh City Open University, Ho Chi Minh City, Vietnam; University of Pitesti, Romania; Institute of Doctoral and Post-doctoral Studies, University Lucian Blaga of Sibiu, ROMANIA

## Abstract

The sustainable development goal seems challenging for governments worldwide, including Indonesia, which has faced an ecological deficit due to rapid economic development and population growth since 1999. The study aims to probe the potential asymmetric effects of foreign direct investment and globalization on ecological footprint in Indonesia from 1971 to 2019, which was ignored by previous studies. By adopting the autoregressive distributed lags (ARDL) and nonlinear autoregressive distributed lags (NARDL) approaches, the results clearly reveal that (*i*) The positive shock of globalization has a positive and statistically significant impact on the ecological footprint; (*ii*) the impact of foreign direct investment on the ecological footprint is asymmetric in the long run. Accordingly, the study found that the influence of negative changes in foreign direct investment is larger than positive changes. Based on the findings, the study recommends that the Indonesian government carefully consider the long-term consequences of globalization on the environment and reasonable control of foreign direct investment inflows.

## 1. Introduction

Indonesia, one of Southeast Asia’s largest economies, is famous for its abundant natural resources such as timber, oil, and gas. According to Kurniawan and Managi [1], Parker [2], Nathaniel [3], Udemba and Philip [4], Indonesia is an interesting context to explore the relationship between economic activities, human activities, and environmental sustainability. During 1990–2014, Indonesia was considered a country with good wealth per capita, and the growth trend was positively related to biodiversity [3]. The Living Planet Report (LPR) 2014 ranked Indonesia among the top ten countries globally, accounting for over 60% of the total biological capacity of the Earth in 2010. However, pressure to boost economic growth and increase income per person, alongside political instability, has severely harmed the environment in Indonesia. From a surplus ecological footprint country, the Indonesian government has been criticized for not stopping deforestation and forest fires, having rubbish in the streets and rivers, and for poor air quality. The Indonesian government issued several economic policies to boost agricultural development for short-term gain. The rapid expansion of oil palm plantations, along with the ineffectiveness and incoherence of laws and regulations, has led to unexpected outcomes like high deforestation rates, soil erosion, loss of biodiversity, and related issues. Parker [2], Wibisana [5] noted that Indonesia’s environmental problems are many and dire. It is not only air pollution but also water quality in Indonesia’s rivers, which is alarming. Indonesia was listed among the countries in the world’s most polluted rivers. Many marine areas are overfished, with some devoid of fish and other marine species; in some places, local people still fish by blowing up coral reefs (with explosives), reducing them to rubble. Hence, Indonesia’s key current challenge is balancing its economic development with the need to protect the environment [1, 5, 6].

Some economists such as Shahzad, Ferraz et al. [7], and Usman, Akadiri and Adeshola [8] advised that expanding globalization and enhancing foreign direct investment inflows may help reduce environmental problems. Globalization has accelerated economic growth worldwide and significantly influenced political, socioeconomic, and environmental facets of daily life [9, 10]. Globalization has facilitated advancements in technology, transportation, and communication, which have made it easier and faster to conduct business and exchange information across distances. As a result, globalization will enhance economic growth, job creation, and poverty reduction in some world regions. Ahmed, Zhang and Cary [11] showed that the connectivity between countries increases the transfer of technologies, reduces energy consumption, and encourages the use of environment-friendly technologies, which in turn improves the environment. Similarly, foreign direct investment (FDI), as a key component of globalization, has enabled multinational corporations to expand their operations beyond their home countries and tap into new markets [12–14]. In recent decades, globalization has led to an increase in FDI flows and has created opportunities for businesses and economies to grow. FDI can positively contributes to sustainable development by supporting research and development activities in manufacturing and infrastructure development [15, 16]. Multinational enterprises often use advanced technologies and best practices. This can lead to adopting cleaner and more efficient technologies, reducing the environmental impact of production processes [17]. Moreover, many multinational companies adhere to strict environmental management standards in their home countries. When these standards are applied to their operations in host countries, they can contribute to improved environmental practices and reduce the ecological footprint [18].

In contrast, several economists and researchers [19, 20] have noted that the rapid expansion of economic activities has also resulted in adverse environmental impacts, as evidenced by the increasing severe ecological deficit caused by human and economic activities. Previous studies revealed that the relationship between globalization, FDI, and ecological footprint is complex and multifaceted [21–23]. On the one hand, globalization and FDI can create opportunities for technology transfer, knowledge exchange, and investment in sustainable development practices, which may help to reduce the ecological footprint. On the other hand, they can also contribute to increased consumption, resource depletion, and pollution, which may exacerbate the ecological footprint. Adeel-Farooq, Riaz and Ali [24] noted that the positive or negative impact of FDI on the ecological footprint depends on the policies and practices adopted by both the host country and the foreign investors. It means that FDI can contribute to environmental quality in a host country if it has strict environmental regulations and vice versa. Therefore, examining how globalization and FDI affect ecological footprint and identifying potential policy measures to mitigate negative impacts and promote sustainable development is essential [25–27].

The relationship between globalization, FDI, and waste harmful to the environment in Indonesia has received much attention because it is a country that has been rapidly developing in recent years and has become increasingly connected to the global economy. Having faced two consecutive crises—the Asian financial crisis in 1997 and the global financial crisis in 2008—Indonesia witnessed a sharp decline in foreign direct investment and challenges related to globalization, economic instability, a devalued currency, and political uncertainty. However, since 2010, Indonesia has seen a gradual increase in FDI, driven by factors such as economic stability, natural resource opportunities, and a growing consumer market. The country continued to liberalize its investment policies during this period. Indonesia also continues to embrace globalization, participating in regional economic initiatives and trade agreements. These events, combined with the bleak picture of the current environmental situation, raise doubts about the rise in FDI and how globalization may cause unexpected problems in Indonesia’s environment.

Compared to available studies for Indonesia, the contributions of this study will be presented below. *First*, the study uses an ecological footprint index instead of conventional emissions indicators because ecological footprints can also provide insights into the long-term sustainability of human activities and the potential for future generations to meet their needs [28, 29]. While important, gases such as CO_2_, SO_2_, and NO_2_ are often reactive and do not necessarily reflect the long-term consequences of human activities on the environment [30]. *Second*, the authors employ autoregressive distributed lag (ARDL) and nonlinear autoregressive distributed lag (NARDL) approaches to examine the extended connections between globalization, FDI, and ecological footprint from 1971 to 2019. The concurrent application of these approaches serves as a robust check for the findings. The ARDL approach is adept at handling linear relationships, whereas NARDL reveals differences in the responses to positive and negative changes and how these changes occur in the short and long term. Ahmed, Cary and Le [31] argued that the policy implications based on a linear framework are unrealistic if the variables have nonlinear properties. Hence, by juxtaposing the outcomes, the study can assess which approach better aligns with the dataset, evaluate the findings, and provide an in-depth understanding of the short- and long-run interactions, especially asymmetric effects. *Third*, the study selects Indonesia as the research background because, in the past, Indonesia was one of the leading countries with high biological capacity in the world, but this situation has disappeared. Currently, the ecological footprint in Indonesia is less than the average biocapacity of the world. What is the cause of this? Is increasing globalization and FDI the cause of this problem? Can negative and positive changes in FDI attraction and globalization lead to effects of different magnitude or direction on the ecological footprint? These questions will be answered in this article.

## 2. Literature review

### 2.1. The literature on globalization and ecological footprint

Globalization has sparked economic growth, significantly impacting human life’s political, environmental, and socioeconomic facets [32, 33]. Globalization refers to increased interconnectedness and interdependence among countries, economies, and people worldwide. It is characterized by the rapid flow of goods, services, capital, and information across borders and the increasing integration of economies and societies [34]. The literature separates globalization into three factors: economic, social, and political globalization [35]. Some studies have concentrated on the effect of globalization on environmental deterioration, but there is no unanimous consensus [36, 37]. Every kind of globalization immediately affects the environment in which people live and work. The endogenous growth theory posits that economic globalization helps countries achieve long-term economic growth while maintaining environmental sustainability [38]. However, implementing environmental policies may harm environmental deterioration or improve environmental quality [39]. Additionally, social globalization accelerates the spread of knowledge, particularly on the finest standards and procedures for conducting business. Promoting green energy sources in economic operations is made easier with knowledge of best practices, which enhances environmental sustainability. Finally, nations that have entered into international agreements and contracts regarding the environment and climate change can adhere to those agreements and contracts [40].

Moreover, globalization impacts environmental sustainability through three effects (scale, composition, and technique effect). For example, globalization’s technique and composition effects encourage using environmentally friendly technologies and machine modifications, which lessens detrimental environmental consequences [11]. However, globalization causes industrialization to raise the demand for energy from various sources like coal and fossil fuels. Primarily, in developing nations with “lax” environmental regulations, globalization frequently promotes the growth of enterprises that produce large amounts of pollution [41]. As industrialization grows, greenhouse gas emissions and global warming endanger environmental quality.

The literature has examined the effects of globalization on the environment using a variety of metrics. Grossman and Krueger [42] employed the North American Free Trade Agreement (NAFTA) as a proxy to examine the effects of globalization on the environment. They discovered that trade liberalization has scale effects on the environment while controlling for composition and technique influence. Sabir and Gorus [34] used an autoregressive distributional lag (ARDL) model to examine the effects of economic globalization and technological advancements on environmental degradation in South Asian nations between 1975 and 2017. Researchers applied FDI, trade openness, and the KOF economic globalization index as measures of globalization. They investigated an inverted U-shaped relationship between globalization, technical advancements, and environmental deterioration, supporting the existence of EKC in South Asian nations. These outcomes showed that indicators of globalization, including FDI, trade openness, and the KOF index have a favorable and statistically significant impact on ecological footprint.

Ahmed, Wang et al. [32] found the nexus between globalization and ecological footprint in Malaysia from 1971 to 2014. The results showed that although globalization does not considerably influence the ecological footprint, it dramatically raises the ecological carbon footprint. Ashraf [43] emphasized globalization and modernization, encouraging bilateral cooperation and strategic connectivity among countries. Using the Generalized Method of Moments, he argued that globalization increased the ecological footprint in the 75 Belt and Road Initiative countries between 1984 and 2019. Similarly, applying the dynamic heterogeneous panel estimation approaches, Lv and Xu [44] demonstrated that a 1% rise in economic globalization results in a 0.11 percent reduction in CO_2_ emissions in 15 nations during the period of 1970–2012.

In contrast, Rudolph and Figge [45] found that political globalization did not affect ecological footprint across 146 nations. Nevertheless, they discovered that although social globalization lessens the ecological footprint, economic globalization increases it. Zaidi, Zafar et al. [46] investigated the association between financial development, globalization, and CO_2_ emissions for Asia Pacific Economic Cooperation (APEC) economies from 1990 to 2016. They applied Continuously Updated Bias-Corrected (Cup-BC) and Continuously Updated Fully Modified (Cup-FM) techniques and concluded that during this time, the environmental quality of APEC countries improved due to these factors. Majeed, Wang et al. [47] agreed that economic globalization also mitigates emission levels in the GCC economies when the study applied a cross-sectional autoregressive distributed lags (CS-ARDL) estimator.

### 2.2. The literature on foreign direct investment (FDI) and ecological footprint

Foreign direct investment (FDI) has been recognized as essential for countries to promote sustainable economic growth and impacts many macroeconomic issues [48]. Foreign direct investment (FDI) is the result of cross-border investments made by citizens (including individuals and businesses) of a home nation to acquire a long-term interest (often at least 10% of the ownership) in a company operating in another (host) country [49]. Furthermore, a major benefit of FDI is facilitating the transfer of knowledge, technology, management know-how, and financial capital from the home country to the host country [25]. Although many theories have explained the connection between FDI and ecological footprints, the Pollution Haven and Halo hypotheses are the most prominent. These two theories show contrasting explanations for the relationship between FDI and environmental quality.

On the one hand, the negative impact is confirmed, meaning that focusing on increasing FDI will harm environmental sustainability or increase emissions into the environment. FDI is explained by the pollution haven hypothesis, which suggests that FDI is more harmful to ecology in developing countries than in developed countries. The Pollution Haven Hypothesis is a theory that suggests that industries relocate to countries with less stringent environmental regulations, where they can produce goods at a lower cost due to lower compliance costs. This hypothesis assumes that environmental regulations raise production costs, and companies seek to avoid these costs by moving their operations to countries with less stringent environmental regulations. The logic behind the Pollution Haven Hypothesis is that companies will seek to maximize their profits by minimizing costs, and environmental regulations can be a significant cost factor for businesses. By relocating to countries with weaker environmental regulations, companies can avoid the costs associated with complying with stricter environmental regulations [50]. This, in turn, can lead to environmental degradation in the countries where industries relocate. For example, Hakimi and Hamdi [51] discovered bidirectional causality between FDI and CO_2_ emission when conducting a variety of econometric models, including a panel VECM and cointegration. FDI inflows to Morocco and Tunisia are not green FDI damaging the environment.

Alternatively, to place Africa’s FDI flows within the sustainable development framework in the 1980s, Bokpin [52] utilized a 24-year panel data set (1990–2013) throughout Africa to evaluate the influence of FDI inflows on the ecosystem. The combined empirical findings show that increased FDI inflows dramatically worsen environmental deterioration, adversely affecting the sustainability of the environment. According to year dummies, environmental deterioration has increased after 2010, surpassing that of 1990, which served as the reference point. Meanwhile, Adeel-Farooq, Riaz and Ali [24] compared the impact of FDI from industrialized and developing nations on the overall environmental quality of 76 countries between 2002 and 2012. By applying fixed effect estimation, their findings indicated that FDI inflow from industrialized nations enhances the environmental performance of the host nation. However, FDI from developing countries negatively impacts the environmental performance of low- and lower-middle-income host nations. They asserted that the source country’s policy environment, not the host country’s, determines whether foreign direct investment has favorable or negative effects on a host country’s environmental performance. Recognizing this distinction is crucial for developing measures to combat the damaging effects of FDI inflows on the environment. As a result, countries that have suffered harm should impose stronger environmental regulations on FDI from emerging nations.

On the other hand, the pollution-halo theory contends that foreign businesses, particularly those from developed countries, come with more advanced and environmentally friendly technology and management strategies that can enhance the host nation’s environmental quality [20]. The pollution-halo concept is particularly pertinent when local businesses are seen as pollution-intensive compared to global norms. Rahman, Cai and Ahmad [19] examined the relationship between FDI and CO_2_ emissions for the top six Asian nations between 1982 and 2014. The empirical findings showed that in China, Sri Lanka, and India, FDI influx considerably increases CO_2_ emissions in both the long and short run. While FDI has no impact on CO_2_ emissions for Pakistan and the Philippines, it has a considerable adverse impact on Bangladesh. Polloni-Silva, Ferraz et al. [53] demonstrated a negative association between FDI and CO_2_ in the Brazilian So Paulo state. Gao, Pei et al. [54] studied panel data in 14 years (2003–2016) from 19 critical cities in the Sichuan-Chongqing metropolitan agglomeration. The influence of FDI on fine particulate matter (PM_2.5_) pollution and its mechanism of action were considered for both socioeconomic and natural factors using the stochastic impacts by regression on population, affluence, and technology (STIRPAT) model. The findings demonstrated that FDI in the Sichuan-Chongqing urban agglomeration had validated the “pollution halo” idea, which means the introduction of FDI helps reduce PM_2.5_ pollution.

To our best knowledge, despite the abundance of previous studies [1, 3, 55, 56] about factors affecting environmental problems in Indonesia, some questions about the nature of the impact of FDI and globalization on ecological footprint in Indonesia are not fully explained. A significant weakness of these studies is that they assume the impact of FDI, globalization, economic growth, and energy consumption on ecological footprint is symmetric. Recently, many studies have confirmed that a large number of macroeconomic variables incorporate non-linear properties, for example, financial development [57], tourism development [58, 59], and energy consumption [60, 61]. Hence, these raise concerns that a linear framework can not fully explain the impact of FDI and globalization on ecological footprint, and that the effectiveness of policy implications based on this framework is unreliable. Moreover, the severe ecological deficit in Indonesia can be directly and indirectly based on human capital development and economic growth. Individuals can modify their consumption lifestyle, reduce waste, use renewable energy, and plant more trees, which in turn influence their ecological footprint [26, 62]. Therefore, by integrating four macroeconomic variables, including FDI, globalization, economic growth, and human capital, the study aims to draw a more comprehensive picture regarding how FDI and globalization are related to ecological footprint in Indonesia and focuses on exploring their potential asymmetric effects.

## 3. Research model and methodology

### 3.1. Research model and data source

The literature review section showed the links between EF and other macroeconomic variables, including economic growth, human capital, foreign direct investment, and globalization. Many studies [4, 6, 63] investigated the impacts of FDI and international trade on environmental degradation in Indonesia. However, whether this relationship is symmetric or asymmetric has not been settled. Therefore, to probe the potential asymmetric effects of FDI and globalization on EF, the initial model is proposed as follows:

$$\log EF_{t}=\beta_{0}+\beta_{1}.\log GDP_{t}+\beta_{2}.HC_{t}+\beta_{3}.Global_{t}+\beta_{4}.FDI_{t}+\varepsilon_{t}$$ (Eq 1)

where *t* is time (from 1971 to 2019), and *u*_*t*_ is an error term. *EF* is the ecological footprint index (units: gha per person) and was collected from the Global Footprint Network. *logGDP* is the logarithm of income per capita (U.S. dollars, at the fixed price 2010), while *FDI* is foreign direct investment per capita (U.S. dollars). Both GDP and FDI variables were taken from the World Bank database. *HC* is the index of human capital per person (units: points) and was collected from the Federal Reserve Bank of St. Louis. Moreover, *Global* is the globalization index (units: points), and the database was collected from the Swiss Economic Institute. After 2019, Indonesia’s human capital per capita index has not been calculated and announced. Thus, the database’s range of this study is from 1971 to 2019.

### 3.2. Econometric strategy

The study applies the ARDL and NARDL approaches based on their advantages. In comparison with classical regression, some advantages of the ARDL and NARDL approaches are given: (*i*) They allow them to capture relationships between both stationary and non-stationary variables; (*ii*) They enable the simultaneous estimation of both long- and short-run symmetries/asymmetries, providing a comprehensive analysis of the data, and avoiding biased findings [64–66].

Accordingly, to investigate the symmetric association among variables in the model, the work applies the ARDL approach, and Eq (1) is written by the ARDL(p,q) approach as:

$$\begin{array}{l} \Delta \log EF_{t}=\beta_{0}+\beta_{1}\log EF_{t-1}+\beta_{2}\log GDP_{t-1}+\beta_{3}HC_{t-1}+\beta_{4}Global_{t-1}+\beta_{5}FDI_{t-1}+\\ +\sum_{j=1}^{p-1}\alpha_{1j}\Delta \log EF_{t-j}+\sum_{j=0}^{q}\alpha_{2j}\Delta \log GDP_{t-j}+\sum_{j=0}^{q}\alpha_{3j}\Delta HC_{t-j}+\\ +\sum_{j=0}^{q}\alpha_{4j}\Delta Global_{t-j}+\sum_{j=0}^{q}\alpha_{5j}\Delta FDI_{t-j}+\varepsilon_{t} \end{array}$$ (Eq 2)

where, Δ is the first difference, and *ɛ*_*t*_ is an error term. Furthermore, *β*_*i*_ (*i* = 1 to 5) denotes the coefficient of long-run impact, while *α*_*i*_ (*i* = 1 to 5) is the coefficient of short-run impact. Moreover, *p* and *q* are the optimal lag length of each variable.

However, the ARDL approach ignored a potential asymmetric effect of interested variables. The study followed the suggestion of Shin, Yu and Greenwood-Nimmo [67] and applied the nonlinear ARDL approach to Eq(1) to overcome this limitation. To explore the potential asymmetric effect of the FDI variable on the EF, Eq (1) is written by the NARDL(p,q) approach as follows:

$$\begin{array}{l} \Delta \log EF_{t}=\beta_{0}+\beta_{1}\log EF_{t-1}+\beta_{2}\log GDP_{t-1}+\beta_{3}HC_{t-1}+\beta_{4}Global_{t-1}+\beta_{5}^{+}FDI_{t-1}+\beta_{5}^{-}FDI_{t-1}+\\ +\sum_{j=1}^{p-1}\alpha_{1j}\Delta \log EF_{t-j}+\sum_{j=0}^{q}\alpha_{2j}\Delta \log GDP_{t-j}+\sum_{j=0}^{q}\alpha_{3j}\Delta HC_{t-j}+\sum_{j=0}^{q}\alpha_{4j}\Delta Global_{t-j}+\\ +\sum_{j=0}^{q}\alpha_{5j}^{+}\Delta FDI_{t-j}+\sum_{j=0}^{q}\alpha_{5j}^{-}\Delta FDI_{t-j}+\varepsilon_{t} \end{array}$$ (Eq 3)

where, $\beta_{5}^{+}$ and $\beta_{5}^{-}$ denotes the long-run asymmetric coefficients of the positive and negative changes in FDI, and $\alpha_{5}^{+}$ and $\alpha_{5}^{-}$ are the short-run asymmetric coefficients. The cumulative function of positive and negative changes in FDI is structured as:

$$\begin{array}{l} FDI_{t}^{+}=\sum_{j=1}^{t}\Delta FDI_{j}^{+}=\sum_{j=1}^{t}\max(\Delta {\mathrm{FDI}}_{j},0)\\ FDI_{t}^{-}=\sum_{j=1}^{t}\Delta FDI_{j}^{-}=\sum_{j=1}^{t}\min(\Delta FDI_{j},0) \end{array}$$

The Wald test is applied to verify the asymmetric effect of FDI variable in the short- and long-term. The null hypothesis of short-run asymmetric coefficient is specified as follows:

$H_{0,SR}:\sum_{j=0}^{q}\alpha_{5j}^{+}=\sum_{j=0}^{q}\alpha_{5j}^{-}$ against the alternative hypothesis $H_{1,SR}:\sum_{j=0}^{q}\alpha_{5j}^{+}=\sum_{j\neq 0}^{q}\alpha_{5j}^{-}$ Similarly, the null hypothesis of long-run asymmetric coefficient is given as:

$H_{0,LR}:\beta_{5}^{+}=\beta_{5}^{-}$ against the alternative hypothesis $H_{1,LR}:\beta_{5}^{+}\neq \beta_{5}^{-}$ If the Wald test is significant, it is evidence to reject the null hypothesis, implying that FDI has asymmetric effects on ecological footprint. The asymmetric cumulative dynamic multiplier effects of a unit change in FDI on EF are specified:

$$m_{h}^{+}=\sum_{j=0}^{h}\frac{\partial \log EF_{t+j}}{\partial FDI_{t}^{+}};m_{h}^{-}=\sum_{j=0}^{h}\frac{\partial \log EF_{t+j}}{\partial FDI_{t}^{-}}\;\mathrm{and}\;h=0,1,2\ldots .$$

Note that as h→∞ then $m_{h}^{+}\to \beta_{5}^{+},m_{h}^{-}\to \beta_{5}^{-}$, where $\beta_{5}^{+}$ and $\beta_{5}^{-}$ are the asymmetric long-run coefficients, respectively.

We also use similar logic to identify the asymmetric effects of globalization on ecological footprint in Indonesia. The positive and negative shocks of globalization refer to the potential consequences of stimulating or reducing the degree of globalization on ecological footprint. Globalization has been credited with many positive effects, such as increased trade and economic growth, but there are also concerns about its negative effects, such as increased inequality, job losses, and environmental degradation [24, 25]. Additionally, the study employs more diagnostic tests, including normality, autocorrelation, heteroscedasticity, the cumulative sum of recursive residuals (CUSUM), and the sum of square recursive residuals (CUSUMSQ) tests to confirm that the initial model is stable. The findings will prove how foreign direct investment and globalization are related to the ecological footprint to aid in building more practical and successful sustainable development policies for Indonesia.

## 4. Empirical results

### 4.1. Descriptive statistics

Fig 1 captures the dynamic of our variables, where it reveals that four variables increase between 1971–2019. The graph also shows that the FDI per person has substantial volatility in the same period. More precisely, there was a wave of multinational enterprises retreating in Indonesia due to political turmoils between 1998 and 2003. Table 1 reports the descriptive statistics of variables. The lowest value of *logEF*, *logGDP*, *HC*, *FDI*, and *Global* variables are 0.043; 6.690; 1.371; -21.42; and 30.67, respectively, while the highest value is 0.536; 8.401; 2.417; 88.25, and 64.25.

**Fig 1:** Plots of the volatility of variables by authors.

**Table 1:** The descriptive statistic of variables.

Indicators	*logEF*	*logGDP*	*HC*	*Global*	*FDI*
Mean	0.266	7.570	1.969	50.39	19.94
Median	0.278	7.641	2.035	50.92	5.99
Maximum	0.536	8.401	2.417	64.25	88.25
Minimum	0.043	6.690	1.371	30.67	-21.42
Std. deviation	0.145	0.481	0.356	10.92	29.20
Observations	49	49	49	49	49

### 4.2. Unit root tests

According to Pesaran and Shin [65] and Shin, Yu and Greenwood-Nimmo [67], the condition to apply the ARDL and NARDL approaches is that all examined variables should not be stationary at the second difference I(2). To verify this, the study used a popular ADF test proposed by Dickey and Fuller [68], and a nonlinear KSS test introduced by Kapetanios, Shin and Snell [69] to confirm the level of stationarity of the variables. The outcomes in Table 2 reveal that three variables (*logEF*, *logGDP*, *Global*) in our model are stationary at the first difference I(1). The ADF test has provided an unclear conclusion regarding the HC and FDI variables. However, the KSS test confirmed that both these variables are stationary at the first difference.

**Table 2:** The results of unit root tests.

Variables	Level		First difference	
	ADF test	Nonlinear (KSS) test	ADF test	Nonlinear (KSS) test
***logEF***	-3.268	0.204	-7.784***	-2.286*
***logGDP***	-2.637	0.514	-5.086***	-2.971**
***HC***	-0.364	-2.013	-1.777	-2.176*
***Global***	-1.198	-0.345	-5.699***	-3.111**
***FDI***	-2.633	-1.159	-3.023	-5.319***

Note

***, **, and * significant at 1%, 5% and 10%, respectively.

The study also used the well-known BDS independence test introduced by Broock, Scheinkman et al. [70] to assess the nonlinearity properties of each variable. Table 3 reveals that the computed variables are not distributed uniformly and independently. It also suggests that nonlinear property exists in the observed values, and the condition for applying the NARDL approach is satisfied [71].

**Table 3:** The BDS test.

Variables	Dimension	BDS statistics	SD	z-stats	Prob
*logEF*	2	0.1606	0.0067	23.912	0.000
	3	0.2635	0.0107	24.478	0.000
	4	0.3222	0.0129	24.928	0.000
	5	0.3595	0.0136	26.476	0.000
	6	0.3945	0.0132	29.884	0.000
*logGDP*	2	0.2001	0.0063	31.503	0.000
	3	0.3376	0.0102	33.129	0.000
	4	0.4342	0.0122	35.463	0.000
	5	0.5027	0.0128	39.038	0.000
	6	0.5525	0.0125	44.098	0.000
*HC*	2	0.2079	0.0069	29.918	0.000
	3	0.3517	0.0111	31.614	0.000
	4	0.4510	0.0133	33.801	0.000
	5	0.5204	0.0140	37.155	0.000
	6	0.5685	0.0136	41.787	0.000
*Global*	2	0.1910	0.0063	30.332	0.000
	3	0.3162	0.0100	31.556	0.000
	4	0.4002	0.0119	33.511	0.000
	5	0.4584	0.0124	36.803	0.000
	6	0.4968	0.0120	41.334	0.000
*FDI*	2	0.1116	0.0147	7.563	0.000
	3	0.1901	0.0239	7.949	0.000
	4	0.2318	0.0291	7.978	0.000
	5	0.3068	0.0309	9.924	0.000
	6	0.3132	0.0304	10.287	0.000

### 4.3. Cointegration test

Another condition for applying the ARDL and NARDL approaches is that there is a cointegration among the variables in the long run [65]. To identify this, the Bound test proposed by Pesaran, Shin and Smith [71] was used, with the null hypothesis that H_0_: *β*_*1*_ = *β*_*2*_ = *β*_*3*_ = *β*_*4*_ = *β*_*5*_ = 0, against the alternative hypothesis H_1_: *β*_*1*_ ≠ *β*_*2*_ ≠ *β*_*3*_ ≠ *β*_*4*_ ≠ *β*_*5*_ ≠ 0. The empirical results in Table 4 showed that the value of F-statistic is 5.640 and 8.026 in symmetric and asymmetric analysis, respectively. These values are greater than the critical value of the upper bound (= 5.173) at the level of 1% significant. It is evidence to reject the null hypothesis, implying that our data series is integrated and the second condition for applying the ARDL and NARDL approaches is satisfied [58, 65].

**Table 4:** Bound test for ARDL and NARDL approaches.

F-Bounds test		Null hypothesis: No level relationship		
Test statistic	Value	Signif	I(0)	I(1)
F-statistic for ARDL model	** **5.640	5%	2.850	3.905
k	4	1%	3.892	5.173
F-statistic for NARDL model	8.026	5%	2.618	3.863
k	4	1%	3.505	5.121

### 4.4. Symmetric and asymmetric effect analysis

After all conditions of the ARDL and NARDL approaches are met, the study employs two approaches to explore the symmetric and asymmetric effects of foreign direct investment, and globalization on ecological footprint in Indonesia. Table 5 reports the symmetric outcomes, while Table 6 presents the asymmetric results.

**Table 5:** The symmetric ARDL findings.

Dependent variable: Δ*logEF*			
Variables	Coefficient	Standard error	T-ratio [Prob]
*CointEq(-1)*	-0.569	0.107	-5.33 [0.000]
*logGDP(-1)*	0.134	0.048	2.82 [0.008]
*HC*	-0.039	0.056	-0.70 [0.487]
*Global(-1)*	0.003	0.001	1.88 [0.068]
*FDI(-1)*	0.001	0.000	1.48 [0.147]
Δ*logGDP*	0.331	0.113	2.92 [0.006]
Δ*FDI(-1)*	-0.001	0.000	-2.47 [0.019]
Δ*Global*	0.003	0.003	1.34 [0.188]
Δ*Global(-1)*	-0.004	0.002	-1.62 [0.116]
Δ*Global(-2)*	-0.004	0.002	-1.56 [0.126]
*Intercept*	-0.9488	0.284	-3.34 [0.002]
R^2^	0.6161	R^2^-adj	0.4765
$\chi_{SC}^{2}$	2.156 [0.133]	$\chi_{FF}^{2}$	2.336 [0.136]
$\chi_{NORM}^{2}$	0.403 [0.817]	$\chi_{HET}^{2}$	1.883 [0.075]
CUSUM test	Stable	CUSUMSQ	Stable

$\chi_{SC}^{2}$, $\chi_{FF}^{2}$, $\chi_{NORM}^{2}$, $\chi_{HET}^{2}$ denotes LM tests for serial correlation, functional form, normality, and heteroskedasticity, respectively. The value in brackets is the corresponding p-value.

**Table 6:** The asymmetric ARDL findings.

Dependent variable: Δ*logEF*			
Variables	Coefficient	Standard error	T-ratio [Prob]
*CointEq(-1)*	-0.7276	0.133	-5.47 [0.000]
*logGDP(-1)*	0.2598	0.058	4.50 [0.000]
*HC(-1)*	-0.2619	0.116	-2.25 [0.035]
*Global* ^*+*^ *(-1)*	0.0080	0.002	2.88 [0.009]
*Global* ^*-*^ *(-1)*	0.0046	0.008	0.54 [0.589]
*FDI* ^*+*^ *(-1)*	0.0009	0.000	2.36 [0.028]
*FDI* ^*-*^ *(-1)*	0.0011	0.001	2.06 [0.053]
Δ*logEF(-1)*	-0.2820	0.133	-2.13 [0.046]
Δ*logGDP*	0.4512	0.107	4.21 [0.000]
Δ*HC(-1)*	-0.3706	0.708	-0.51 [0.606]
Δ*Global*^*+*^	0.0066	0.004	1.52 [0.144]
Δ*Global*^*-*^	-0.0008	0.006	-0.13 [0.879]
Δ*FDI*^*+*^	-0.0000	0.000	-0.08 [0.935]
Δ*FDI*^*-*^	0.0006	0.000	1.15 [0.263]
*Intercept*	-1.4686	0.344	-4.25 [0.000]
R^2^	0.8424	R^2^-adj	0.6532
$\chi_{SC}^{2}$	3.241 [0.063]	$\chi_{FF}^{2}$	2.709 [0.116]
$\chi_{NORM}^{2}$	2.115 [0.347]	$\chi_{HET}^{2}$	0.539 [0.925]

Note: The superscripts “+” and “-” present the cumulative function of positive and negative changes, respectively. $\chi_{SC}^{2}$, $\chi_{FF}^{2}$, $\chi_{NORM}^{2}$, $\chi_{HET}^{2}$ denotes LM tests for serial correlation, functional form, normality, and heteroskedasticity, respectively. The value in brackets is the corresponding p-value.

According to Table 5, the coefficient of CointEq(-1) variable is -0.569 and significant at the level of 1%, which implies that the ecological footprint index could re-adjust to the long-run equilibrium after the short-run shocks caused by globalization, FDI, economic growth, or human capital. Table 5 also reports that economic growth (*β* = 0.134, *p-value* = 0.008) and globalization (*β* = 0.003, *p-value* = 0.068) variables positively impact EF, implying that an increase in economic growth and expanded globalization lead to an increased ecological deficit in Indonesia. On the contrary, an increase in human capital (*β* = -0.039, *p-value* = 0.487) leads to a decrease in environmental problems, but this conclusion is not significant. Besides, the symmetric result has failed to indicate that FDI (*β* = 0.001, *p-value* = 0.147) is related to ecological footprint. This result implies that the ADRL approach may not be appropriate for evaluating the determinants of ecological footprint in Indonesia and could provide a biased result.

To overcome the limitation of ARDL approach, the study utilized the NARDL method. In the long-run, Table 6 shows that the impact of economic growth (*β* = 0.2598, *p-value* = 0.000) on EF is positive and significant. Accordingly, a 1% increase in income per capita leads to a 0.2598% increase in ecological footprint. In addition, human capital negatively influences ecological footprint in the long term (*β* = -0.2619, *p-value* = 0.035), but it does not affect it in the short run. However, the main aim of the study is to explore the potential asymmetric effects of FDI, and globalization on EF. The empirical results in Table 6 reveal that the positive changes in globalization positively influence EF (*β* = 0.008, *p-value* = 0.009), while the impact of negative changes is unclear (*β* = 0.0046, *p-value* = 0.589). The Wald test results in Table 7 reveal that the null hypothesis of asymmetric effect, in the long run, is rejected and accepted in the short run. These findings allow us to conclude that the impact of globalization on EF in Indonesia is symmetric in the short run but asymmetric in the long run. More precisely, the influence of positive changes (= 0.008) in globalization is greater than negative changes (= 0.0046), and enhancing the degree of globalization stimulates the ecological deficit in Indonesia.

**Table 7:** The Wald test results.

Variables	*Short-run Wald test*	*p-value*	*Long-run Wald test*	*p-value*
*Global*	3.6584	0.1605	8.7771	0.0092
*FDI*	1.8292	0.1864	7.8643	0.0196

Similarly, Table 6 also showed that boosting FDI attraction might reduce the ecological deficit in the short term, but stimulate environmental deterioration in the long term (*β* = 0.0009, *p-value* = 0.028). The Wald test in Table 7 documents that the null hypothesis is rejected in the long run but is accepted in the short run. These findings imply that the influence of FDI on EF in Indonesia is asymmetric in the long term, and the impact of a negative shock (= 0.0011) in FDI on EF is greater than that of a positive shock (= 0.0009).

Furthermore, all diagnostic tests are satisfied, including normality, autocorrelation, heteroscedasticity, the cumulative sum of recursive residuals (CUSUM), and the sum of square recursive residuals (CUSUMSQ) tests. Figs 2 and 3 demonstrate that, at the level of 5% significance, the blue lines representing CUSUM and CUSUMSQ are within the critical bound (indicated by red lines). These findings allow the study to conclude that the proposed model is stable. Fig 4A and 4B graph the dynamic impacts of positive and negative changes in globalization and FDI. These results further imply that just observing in a linear framework for factors of globalization and FDI would be prone to produce misleading and biased results.

**Fig 2:** The CUSUM plot.

**Fig 3:** The CUSUMSQ plot.

**Fig 4:** a. The dynamic multiplier graphs of Global. b. The dynamic multiplier graphs of FDI.

### 4.5. Robustness

The study also employed three other approaches, including fully modified ordinary least squares (FMOLS), dynamic ordinary least squares (DOLS), and canonical cointegrating regression (CCR) to robustness. Outcomes are presented in Table 8. Accordingly, the three approaches reveal similar direction and margin impact results. It is also in line with the findings of the NARDL approach. Hence, this evidence allows the study to conclude that empirical outcomes are reliable and can be used to suggest policy implications for Indonesia’s economy.

**Table 8:** The FMOLS, DOLS, CCR results.

Variables	Approaches	Coefficient	Standard error	T-ratio [Prob]
*logGDP*	FMOLS	0.1822	0.067	2.70 [0.009]
*HC*		-0.0867	0.101	-0.86 [0.394]
*Global*		0.0060	0.003	2.17 [0.036]
*FDI*		0.0009	0.001	2.31 [0.025]
*Intercept*		-1.2603	0.368	-3.42 [0.001]
*logGDP*	DOLS	0.2317	0.080	2.88 [0.007]
*HC*		-0.0147	0.159	-0.09 [0.926]
*Global*		0.0023	0.004	0.51 [0.616]
*FDI*		0.0002	0.001	0.25 [0.805]
*Intercept*		-1.5417	0.446	-3.45 [0.001]
*logGDP*	CCR	0.1857	0.068	2.71 [0.009]
*HC*		-0.0925	0.101	-0.91 [0.365]
*Global*		0.0060	0.003	2.19 [0.034]
*FDI*		0.0009	0.001	2.13 [0.039]
*Intercept*		-1.2775	0.374	-3.41 [0.001]

### 4.6. Discussion

The empirical findings uncover fascinating insights regarding the influence of foreign direct investment and globalization on Indonesia’s ecological footprint. These results highlight that while efforts to attract FDI might initially alleviate the ecological deficit in the short run, it eventually leads to environmental decay in the long term. This suggests that the initial positive impact on the environment is not sustainable, and the long-term consequences of FDI on the environment are considerably more harmful. Additionally, these findings indicate an asymmetric relationship between FDI and ecological footprint in Indonesia, where a negative shock to FDI has a greater impact on ecological footprint than a positive shock. This asymmetry implies that the environmental effects of a reduction in FDI are greater than those of an increase in FDI. Furthermore, these findings lend support to the pollution haven hypothesis, which posits that countries, particularly those in the middle-income bracket like Indonesia, may experience a negative impact on their environment due to foreign direct investment (FDI). This aligns with the empirical results presented by Doytch [72] when Indonesia belongs to the group of middle-income countries that tend to be negatively affected by FDI. Similar results were also found in Solarin, Al-Mulali et al. [73], Wagner and Timmins [74].

According to Doytch [72], several factors contribute to this phenomenon, including the types of industries attracted by FDI, existing regulatory frameworks, and the country’s overall environmental policies. As per the Investment Law, specifically Law Number 25 of 2007 on Capital Investment amended by the Omnibus Law, investors have two options for engaging in business activities in Indonesia through foreign direct investment. They can either establish a new PT PMA (Perseroan Terbatas Penanaman Modal Asing or Limited Liability Company with Foreign Direct Investment) or acquire an existing company within the country [75, 76]. Having foreign investment in the form of a PT PMA allows for greater regulatory oversight by Indonesian authorities. The regulatory framework for PT PMAs can include a thorough Environmental Impact Assessment (EIA) requirement before project approval [77]. This ensures that potential environmental risks and impacts are thoroughly evaluated and mitigated before a foreign investor can establish or acquire a company. The PT PMA structure provides opportunities for local communities to engage with foreign investors during the establishment or acquisition process. This engagement can lead to a better understanding of local environmental concerns, allowing for incorporating community feedback into environmental protection plans. In terms of acquiring existing companies, the government imposes a form of accountability on foreign investors for the environmental practices of those companies. This can lead to a more immediate and direct impact on improving environmental performance. Additionally, the acquisition process allows for faster implementation of environmental improvements compared to starting from scratch. Foreign investors can implement changes and upgrades more rapidly in existing facilities to align with international environmental standards.

However, this policy also has some disadvantages and challenges related to environmental protection. First, acquiring an existing company may limit the level of control that the government has over its pre-existing environmental practices. Ensuring acquired companies adhere to strict environmental standards may be challenging, especially if they have a history of non-compliance. Second, existing companies may have varying levels of commitment to environmental protection. Some already have robust sustainability practices, while others need significant improvements. The policy may not be uniformly effective in ensuring consistent environmental performance across all foreign-invested entities. Companies may choose locations or industries with less stringent environmental regulations, potentially leading to regulatory arbitrage. This can result in investments being attracted to areas with weaker environmental protection standards, undermining the overall goal of promoting sustainable development. Third, new entrants establishing a PT PMA may face challenges adapting to evolving global environmental standards. The fixed legal structure may not provide the flexibility needed to accommodate emerging best practices in environmental protection. While thorough assessments are essential, prolonged approval processes could discourage foreign investors and hinder the timely implementation of environmentally friendly projects. Fourth, companies may engage in greenwashing, presenting a false image of environmental responsibility to meet regulatory requirements without implementing meaningful, sustainable practices. This can lead to a gap between regulatory compliance and actual environmental impact. To address these disadvantages, policymakers should continuously review and update regulations, strengthen enforcement mechanisms, and consider providing targeted incentives for environmentally friendly investments within the PT PMA framework. Indonesia can implement tiered environmental standards that consider the industry type, size of the investment, and potential environmental impact. This allows for a nuanced approach, ensuring that smaller-scale investments with lower environmental footprints are subject to appropriate, yet less burdensome, regulatory requirements.

Moreover, the government should develop targeted incentives for environmentally sustainable investments. These incentives could include tax breaks, reduced import duties on green technologies, and other financial benefits to encourage companies to adopt and invest in eco-friendly practices. Besides, fostering collaboration between the government, private sector, and civil society to promote sustainable business practices is necessary. Public-private partnerships can facilitate information sharing, joint initiatives, and the development of industry-specific sustainability standards. This information is vital for policymakers as they strive to strike a balance between attracting foreign investments and safeguarding the environment. Understanding the long-term repercussions of FDI on the environment allows for developing more sustainable and effective policies that align economic development goals with environmental conservation efforts.

The findings also indicate that only positive changes in globalization have a positive and statistically significant impact on ecological footprint. It means that the positive changes in globalization lead to increased resource exploitation, heightened production and consumption, or other activities contributing to environmental degradation in Indonesia. This suggests that reducing the degree of globalization could help to mitigate ecological deficit in Indonesia and that the impact of globalization on EF is asymmetric in the long term. The above idea has also appeared in Sabir and Gorus [34], Figge, Oebels and Offermans [78] with the context in 171 countries and South Asia, respectively. This finding is particularly relevant given the increasing interconnectedness of the global economy and the potential for global trade and investment to have significant environmental impacts. The remedy involves incorporating various components into positive shifts in globalization, such as enhancing international collaboration on environmental concerns, embracing cleaner technologies, and advocating for sustainable practices in worldwide trade. In these cases, the positive impact on the ecological footprint might mean reducing environmental harm or improving sustainability.

The findings imply that policymakers should thoroughly consider the environmental consequences of foreign direct investment and globalization. It is crucial to devise strategies that effectively minimize the adverse effects. This can be achieved by implementing policies and regulations that effectively curb the environmental impact of FDI. Furthermore, promoting sustainable investment practices and exploring alternative development models that prioritize environmental protection would be beneficial. Additionally, the endeavors to reduce globalization can assist in alleviating the detrimental environmental effects of global trade and investment.

## 5. Conclusion

The asymmetric effects of globalization and foreign direct investment on ecological deficit have been ignored in previous studies in the context of Indonesia. If the nexus between foreign direct investment or globalization and ecological footprint is asymmetric, the policy implications based on symmetric approaches can be unreliable. By adopting the ARDL and NARDL approaches in Indonesia from 1971 to 2019, the empirical results of the study demonstrated some conclusions, as follows:

*Firstly*, the impact of FDI on ecological footprint is symmetric in the short run but asymmetric in the long run. More precisely, FDI stimulates ecological deficit status in the long term, and the influence of negative changes in FDI is greater than positive.

*Secondly*, only positive shifts in globalization positively and statistically significantly influence the ecological footprint. Accordingly, an increase in the degree of globalization leads to an increase in the ecological deficit in Indonesia, and the impact of globalization on EF is asymmetric in the long term.

*Thirdly*, economic growth positively drives EF in Indonesia. Therefore, boosting economic growth can reduce social unrest and create new jobs but exacerbate Indonesia’s ecological deficit.

Based on the empirical result, some policy implications are suggested, as detailed:

*Firstly*, due to structural reforms, Indonesia experienced a 14% rise in foreign investment inflow in 2019, primarily concentrated in the gas, electricity, water, and transportation sectors [4]. The rise in FDI attraction within high energy-consuming sectors has resulted in a decline in environmental sustainability. Particularly, post-1999, the ecological deficit has exceeded the ecological reserve, and this situation is becoming increasingly critical. Faced with the above scenario, the government must evaluate and scrutinize foreign direct investment (FDI) projects in alignment with existing environmentally beneficial policies. For instance, adherence and sustainable development based on the IEA’s Energy Sector Roadmap to Net Zero Emissions in Indonesia should be integral. It is imperative for policymakers to consistently reassess and revise regulations, bolster enforcement mechanisms, and contemplate offering specific incentives for environmentally responsible investments within the PT PMA framework. Indonesia has the potential to establish graduated environmental standards that account for industry type, investment size, and potential environmental consequences. This approach ensures a nuanced strategy, where smaller-scale investments with lower environmental impacts are subjected to fitting and less onerous regulatory requirements.

Additionally, the government should institute targeted incentives to encourage eco-friendly investments, such as tax incentives or subsidies for foreign investors engaged in environmentally friendly projects, such as renewable energy, energy efficiency, and sustainable agriculture. Furthermore, the Indonesian government should replace outdated environmental regulations and implement and enforce stringent environmental standards and regulations to ensure that all businesses, including foreign investors, adhere to sustainable practices [23]. Establishing technology parks or clusters focused on sustainable development to encourage knowledge sharing and collaboration should be considered.

*Secondly*, Indonesia’s policymakers must carefully consider the long-term consequences of globalization on the environment and take decisive action to alleviate its negative effects. By actively promoting renewable energy, implementing policies to reduce waste generation, and promoting recycling, Indonesia can diminish the ecological deficit and forge a path towards a truly sustainable future. In order to counterbalance the adverse consequences of globalization, regulators can foster international collaboration on environmental matters. This entails collaborating with other nations to curb greenhouse gas emissions, safeguard biodiversity, and preserve precious natural resources. Furthermore, Indonesia’s government can play a crucial role in fostering the development of a green economy. Some policies should be considered, such as providing investments in renewable energy [8], innovative green technologies, and sustainable industries.

Furthermore, the Indonesian government should encourage domestic enterprises to foster collaboration between research institutions and businesses to develop and share sustainable technologies and facilitate the international transfer of clean and green technologies. Last but not least, the Indonesian government should establish mechanisms for enforcing environmental standards in global supply chains and encourage cross-cultural understanding of environmental challenges and solutions because international cooperation is essential to address environmental challenges that transcend national borders effectively [22, 79].

Several important findings on the impact of FDI and globalization on environmental quality in Indonesia have been confirmed by this study. However, this work also has its constraints, notably limited data availability. Future research endeavors could enhance their insights by incorporating historical data spanning an extended period to address ecological deficit mitigation. Additionally, while the current research is focused on Indonesia, there is potential for extending its scope to explore analogous issues in various developed and developing economies, aiming to improve our comprehension of the subject. Furthermore, to paint a comprehensive picture of the connection between economic and environmental factors beyond FDI and globalization, it is imperative to delve deeper into research on contributors to the ecological deficit, such as institutional quality and financial development. This would provide a more holistic understanding of the interplay between economic activities and environmental quality.
